# Bidirectional rotating flow of nanofluid over a variable thickened stretching sheet with non-Fourier’s heat flux and non-Fick’s mass flux theory

This article has been retracted.

**DOI:** 10.1371/journal.pone.0265443

**Published:** 2022-04-28

**Authors:** Fazle Mabood, Maria Imtiaz, Maimona Rafiq, Essam Roshdy El-Zahar, Maawiya Ould Sidi, Muhammad Ijaz Khan

**Affiliations:** 1 Department of Information Technology, Fanshawe College, London, ON, Canada; 2 Department of Social and Behavioral Sciences National University of Medical Sciences, Rawalpindi, Pakistan; 3 COMSATS University Islamabad, Attock Campus, District Attock Punjab, Pakistan; 4 Department of Mathematics, College of Science and Humanities in Al-Kharj, Prince Sattam bin Abdulaziz University, Al-Kharj, Saudi Arabia; 5 Department of Basic Engineering Science, Faculty of Engineering, Menoufia University, Shebin El-Kom, Egypt; 6 RT-M2A Laboratory, Mathematics Department, College of Science, Jouf University, Sakaka, Saudi Arabia; 7 Department of Mathematics and Statistics, Riphah International University, Islamabad, Pakistan; Central University of Karnataka, INDIA

## Abstract

The flow of nanofluid over a variable thickened stretching sheet is studied in this article. Non-Fourier’s heat flux and non-Fick’s mass flux are incorporated for heat and mass flow analysis. Silver (*Ag*) and Copper (*Cu*) are considered nanoparticles with water as base fluid. The resulting equations are transformed into the dimensionless form using similarity transformation and solved by RK-4 with the shooting method. The impact of the governing parameters on the dimensionless velocity, temperature, concentration, skin friction coefficient, streamlines, and finally isotherms are incorporated. It is observed that increment in power-law index parameter uplifts the fluid flow, heat, and mass transfer. The increase in the magnitude of skin friction coefficient in (*x-*direction) with wall thickness parameter is high for nanofluid containing silver nanoparticles as compared to copper nanoparticles.

## 1. Introduction

The problem of heat transfer enhancement in engineering and industrial applications is of high priority nowadays. Many applications that require fluid as a cooling agent, such as water, ethylene glycol, and low thermal conductivity oil, limit the heat transfer enhancement. To improve thermal efficiency, new types of fluids such as nanofluids are introduced. Masuda et al. [1] introduced ultrafine particles of Al_2_O_3_, SiO_2_ and TiO_2_ and observed change in thermal diffusivity and fluid viscosity. Nanofluids are described as a mixture composed of dispersed particles of nanometer size in the base fluid; the term initially introduced by Choi [2]. Further, his experimental studies unveiled the fact that the addition of nanoparticles (less than 1% by volume) magnifies the thermal conductivity of the fluid up to approximately two times [3]. Experimental studies of Xuan and Li [4] have shown that the small concentrations of nanoparticles can enhance the thermal conductivity of the suspensions by more than 20%. Akbarinia et al. [5] claimed that nanofluids are more stable and have reasonable viscosity and better properties for wetting, spreading, and dispersing on solid surfaces. Most used base fluids are water, ethylene glycol, and oil, while the common nanoparticles are gold, copper, silver, titanium, and silicon, or their oxides. Nanofluids are extensively used as coolants, lubricants, as well as in practical applications such as cooling and air conditioning, microelectronics, mobile computer processors, and so on. Recently, various researchers studied the behavior and characteristics of nanofluids both experimentally and mathematically. Experimental studies have shown that the addition of nanoparticles in conventional fluids improve the absorption efficiency of solar collectors’ incident radiations (see refs. [6–8]). Also, the important application of nanofluid in microchannel has been discussed in detail by Chamkha et al. [9]. Nanofluids played a very important role in improving heat transfer at nuclear power plants. Because of the high thermal conductivity of the nuclear reactor’s nanofluid heat transfer capacity, it can be a thousand times larger than conventional fluids such as water [10]. Ferrofluids are formed in a liquid carrier by dispersing 10 nm ferromagnetic particles. Recent studies have shown that magnetic nanofluids can be used in many areas of magnetic separation of cells, contrast agent enhancement in magnetic resonance imaging (MRI), magnetic drug targeting, and magnetic hyperthermia (see refs. [11, 12]). Additionally, various researchers have presented mathematical models of nanofluid, among them two are most commonly used. One proposed by Buongiorno [13] and the second by Tiwari and Das [14]. For the comparison between theoretical and experimental data, nanofluid thermal conductivity efficiency is being examined among the models. Various researchers such as [15–21] used Buongiorno’s proposed mathematical nanofluid model [13] which involves the effects of Brownian motion and thermophoresis parameters. The nanofluid model proposed by Tiwari and Das [14] was also employed by several authors such as [22–24].

Recently, the implementation of Cattaneo-Christov model to study the mechanism of heat and mass flux is trending as various researchers adopt this model in problem formulation. The study of heat and mass flux cannot be ignored as the temperature and concentration differences occur within a system or within the systems. In all above-mentioned research, heat and mass transport phenomena are discussed by incorporating classical law of thermodynamics and heat conduction by Fourier [25]. The major drawback of using this law is the restriction of energy and concentration equations to be of parabolic type equations. The physical interpretation of this restriction is that any initial disturbance is rapidly experienced by the medium. Cattaneo [26] in 1948 modified the Fourier law by enforcing a thermal relaxation characteristic time term, called "thermal inertia" which is called Maxwell-Catteneo law. This modified law enables scientists to study heat/mass disturbance through the propagation of finite length wave. But the major difficulty in using this model is the existence of different thermal relaxation times for different materials. Keeping this fact in mind, a very useful time derivative model was developed for the effective heat transfer mechanism by Christov [27]. He replaced the time derivative with Oldroyd upper-convective derivative. The theory, thus, termed as Cattaneo-Christov heat and mass flux theory (CC-model). Haddad [28] investigated the thermal instability while analyzing the flow through Brinkman porous media using CC-model. Imtiaz et al. [29] performed the analysis of two-dimensional flow of non-Newtonian fluid over linearly stretching surface by incorporating the effects thermal relaxation time presented through CC-heat flux model. Mahmood et al. [30] utilized CC-model in heat flux analysis of Casson fluid flow over stretching surface with entropy generation effects. Negative impact of magnetic field on boundary layer flow nanofluid is noticed from the results. Kumar et al. [31] disclosed the influence of CC-model on Reiner-Philippoff flow on stretching surface in the presence of Ohmic heating and transverse magnetic field. Shah et al. [32] presented the effect of CC-heat flux model on Casson ferrofluid flow over the stretching surface in the presence of externally applied magnetic and electric fields. Shah et al. [33] also discussed the impact of CC-model on Darcy-Forchheimer flow of micropolar ferrofluid through porous media. Their study discloses that by increasing electric field strength velocity enhances whereas opposite behavior is noticed for microrotation parameter. Sajid et al. [34] reported the impact of CC-heat flux model on carbon nanotubes for Maxwell velocity slip and Smoluchowski temperature.

The analysis involving Newtonian and non-Newtonian fluid flow over stretched surface finds its application in various engineering processes which involves wire drawing, heat-treated materials travelling between a wind-up roll and a feed role or materials manufactured by extrusion, paper and glass fiber production, cooling of metallic sheets or electronic chips, drawing of plastic sheets, crystal growing, and many others. Final product characteristics depend upon the cooling process in the stretched sheet. This growing interest for studying the stretching sheet flows resulted in numerous research investigations reported in the last two decades. For example, Rubab and Mustafa [35] analyzes the three-dimensional flow of upper convected Maxwell fluid over stretching sheet. They have incorporated the effects of thermal relaxation time and magnetic field to model the problem. Imtiaz et al. [36] performed the study for homogeneous-heterogeneous reactions in MHD radiative flow of second grade fluid due to a curved stretching surface. Zeeshan et al. [37] investigated the numerical study on bi-phase coupled stress fluid in the presence of Hafnium and metallic nanoparticles over an inclined plane. Some considerable mentions can be seen through refs. [33, 38–41]. The investigations cited above focus more on linear stretching surfaces and nonlinearity has been ignored. Although the nonlinear stretching is equally important while discussing the real-life applications of fluid flow. But now the researchers are giving much more attention to this new concept. Therefore, keeping in view the context of non-linearity in stretching rates, recently, Seth and Mishra [42] presented the study dealing with the effects of Navier slip condition and thermal radiation on boundary layer flow of nanofluid generated by nonlinear stretching. Thumma et al. [43] performed numerical investigations on radiative mixed convective boundary layer flow over inclined stretching sheet in the presence of viscous dissipation effects and heat source/sink. Their study closely related to the fabrication of magnetic nanomaterials. Ramya et al. [44] analyzed the effects of slip conditions on boundary layer flow nanofluid over nonlinearly stretching surface. The outcomes of the study reveal that the heat and mass transfer rates are greatly affected by increasing thermal slip condition. Some recent studies can be seen in [45–49].

To our knowledge, nanofluid flow in the regimes of three-dimensional flow and rotating frame over variable thickened stretching sheet has not been explored yet. Purpose of present research is three-fold. Firstly, to formulate the bidirectional flow of silver and copper-water nanofluid bounded by stretching surface with variable thickness in rotating frame of reference. Secondly, to analyze heat and mass transfer with thermal and solutal relaxation effects. And thirdly, to solve the governing non-linear system by applying RK-4 with shooting method. Results are discussed for velocity, temperature, concentration and skin friction coefficients by plotting graphs.

## 2. Mathematical formulation

Here bidirectional flow of an incompressible nanofluid due to a stretching sheet of variable thickness is considered. Thickness of sheet is $z=A(x+y{)}^{\frac{1-n}{2}}$. Copper and silver nanoparticles with water are used as base fluid. We choose the Cartesian coordinate system such that the surface is aligned with the xy-plane and fluid is considered in the space z ≥ 0. The surface is assumed to stretch in the x and y direction with stretching rate c. Also, the fluid rotates with constant angular velocity Ω about the z-axis (see Fig 1). T_w_ is constant wall temperature and T_∞_ is the ambient temperature. Non-Fourier heat flux and non-Fick’s mass flux are taken. The governing equations are

$$\frac{\partial u}{\partial x}+\frac{\partial v}{\partial y}+\frac{\partial w}{\partial z}=0,$$ (1)

$$u\frac{\partial u}{\partial x}+v\frac{\partial u}{\partial y}+w\frac{\partial u}{\partial z}-2\Omega v=\nu_{nf}\frac{\partial^{2}u}{\partial z^{2}},$$ (2)

$$u\frac{\partial v}{\partial x}+v\frac{\partial v}{\partial y}+w\frac{\partial v}{\partial z}+2\Omega u=\nu_{nf}\frac{\partial^{2}v}{\partial z^{2}},$$ (3)

$$\begin{array}{l} u\frac{\partial T}{\partial x}+v\frac{\partial T}{\partial y}+w\frac{\partial T}{\partial z}=\alpha_{nf}\frac{\partial^{2}T}{\partial z^{2}}-\lambda_{E}[u^{2}\frac{\partial^{2}T}{\partial x^{2}}+v^{2}\frac{\partial^{2}T}{\partial y^{2}}+w^{2}\frac{\partial^{2}T}{\partial z^{2}}+2uv\frac{\partial^{2}T}{\partial x\partial y}\\ +2vw\frac{\partial^{2}T}{\partial y\partial z}+2uw\frac{\partial^{2}T}{\partial x\partial z}+\left(u\frac{\partial u}{\partial x}+v\frac{\partial u}{\partial y}+w\frac{\partial u}{\partial z}\right)\frac{\partial T}{\partial x}+\left(u\frac{\partial v}{\partial x}+v\frac{\partial v}{\partial y}+w\frac{\partial v}{\partial z}\right)\frac{\partial T}{\partial y}\\ +(u\frac{\partial w}{\partial x}+v\frac{\partial w}{\partial y}+w\frac{\partial w}{\partial z})\frac{\partial T}{\partial z}], \end{array}$$ (4)

$$\begin{array}{l} u\frac{\partial C}{\partial x}+v\frac{\partial C}{\partial y}+w\frac{\partial C}{\partial z}=D\frac{\partial^{2}C}{\partial z^{2}}-\lambda_{C}[u^{2}\frac{\partial^{2}C}{\partial x^{2}}+v^{2}\frac{\partial^{2}C}{\partial y^{2}}+w^{2}\frac{\partial^{2}C}{\partial z^{2}}+2uv\frac{\partial^{2}C}{\partial x\partial y}\\ +2vw\frac{\partial^{2}C}{\partial y\partial z}+2uw\frac{\partial^{2}C}{\partial x\partial z}+\left(u\frac{\partial u}{\partial x}+v\frac{\partial u}{\partial y}+w\frac{\partial u}{\partial z}\right)\frac{\partial C}{\partial x}+\left(u\frac{\partial v}{\partial x}+v\frac{\partial v}{\partial y}+w\frac{\partial v}{\partial z}\right)\frac{\partial C}{\partial y}\\ +\left(u\frac{\partial w}{\partial x}+v\frac{\partial w}{\partial y}+w\frac{\partial w}{\partial z}\right)\frac{\partial C}{\partial z}]. \end{array}$$ (5)

**Fig 1:** Geometry of the problem.

The corresponding boundary conditions are

$$\begin{array}{l} u=u_{w}=c(x+y{)}^{n},\;v=v_{w}=c(x+y{)}^{n},w=0,T=T_{w},C=C_{w}\;\mathrm{at}\;z=A(x+y{)}^{\frac{1-n}{2}},\\ u\to 0,v\to 0,T\to T_{\infty },C\to C_{\infty }\;\mathrm{as}\;z\to \infty , \end{array}$$ (6)

where *u*, v and *w* depict the velocity components parallel to *x*−, *y*− and *z*−directions, *v* the kinematic viscosity of fluid, *ρ* fluid density, *λ*_*E*_ heat relaxation time and *λ*_*C*_ mass relaxation time. Type of the motion, shape of the surface and behavior of the boundary layer are controlled by the shape parameter *n*. Wall thickness parameter *n* is divided into three cases: the wall thickness parameter decreases for *n*>1, the surface is flat when *n* = 1 and the wall thickness parameter increases for *n*<1. As type of motion is controlled by this parameter so accelerated motion is represented by *n*>1, the linear motion by *n* =0 and the decelerated motion is expressed as *n*<1.

We consider the following transformations

$$\begin{array}{l} \Lambda =\sqrt{\frac{\left(n+1\right)}{2}\frac{c}{\nu_{f}}(x+y{)}^{n-1}}z,u=c(x+y{)}^{n}f^{\prime }(\Lambda ),v=c(x+y{)}^{n}g^{\prime }(\Lambda ),\\ w=-\sqrt{\frac{\left(n+1\right)}{2}c\nu_{f}(x+y{)}^{n-1}}\left[f(\Lambda )+g(\Lambda )+\frac{n-1}{n+1}\Lambda (f^{\prime }(\Lambda )+g^{\prime }(\Lambda ))\right],\\ \theta (\Lambda )=\frac{T-T_{\infty }}{T_{w}-T_{\infty }},\varphi (\Lambda )=\frac{C-C_{\infty }}{C_{w}-C_{\infty }}. \end{array}$$ (7)

Here *μ*_*nf*_, *ρ*_*nf*_, (*ρC*_*p*_)_*nf*_ and *k*_*nf*_ are the effective dynamic viscosity, density, heat capacity and thermal conductivity of the nanofluid [14] which are defined as

$$\mu_{nf}=\frac{\mu_{f}}{(1-\varphi {)}^{2.5}},$$ (8)

$$\rho_{nf}=(1-\varphi )\rho_{f}+\varphi \rho_{s},$$ (9)

$$(\rho C_{p}{)}_{nf}=(1-\varphi )(\rho C_{p}{)}_{f}+\varphi (\rho C_{p}{)}_{s},$$ (10)

$$\frac{k_{nf}}{k_{f}}=\frac{\left(k_{s}+2k_{f})-2\varphi (k_{f}-k_{s}\right)}{\left(k_{s}+2k_{f})+\varphi (k_{f}-k_{s}\right)}.$$ (11)

Here *φ* represents the solid volume fraction of the nanoparticles and the subscripts *s*, *f* and *nf* are used for nano-solid-particles, base fluid, and thermo-physical properties of the nanofluid.

The conservation of mass is fulfilled and Eqs (2–6) are reduced to:

$$\frac{1}{\left(1-\varphi {)}^{2.5}(1-\varphi +\frac{\rho_{s}}{\rho_{f}}\varphi \right)}f^{\prime \prime \prime }+ff^{\prime \prime }+gf^{\prime \prime }-\left(\frac{2n}{n+1}\right)f^{\prime 2}-\left(\frac{2n}{n+1}\right)f^{\prime }g^{\prime }+\frac{4\lambda }{n+1}g^{\prime }=0,$$ (12)

$$\frac{1}{\left(1-\varphi {)}^{2.5}(1-\varphi +\frac{\rho_{s}}{\rho_{f}}\varphi \right)}g^{\prime \prime \prime }+fg^{\prime \prime }+gg^{\prime \prime }-\left(\frac{2n}{n+1}\right)g^{\prime 2}-\left(\frac{2n}{n+1}\right)f^{\prime }g^{\prime }-\frac{4\lambda }{n+1}f^{\prime }=0,$$ (13)

$$\begin{array}{l} \frac{1}{Pr}\frac{k_{nf}}{k_{f}}\frac{1}{\left(1-\varphi +\frac{(\rho c_{p){}_{s}}}{(\rho c_{p{)}_{f}}}\varphi \right)}\theta^{\prime \prime }+f\theta^{\prime }+g\theta^{\prime }+\delta [\frac{(n-1{)}^{2}}{2(n+1)}\{\xi^{2}{f^{\prime }}^{2}\theta^{\prime \prime }+\xi^{2}{g^{\prime }}^{2}\theta^{\prime \prime }-\xi f\prime \prime g\prime \theta \\ -\xi g^{\prime \prime }g^{\prime }\theta^{\prime }+\xi^{2}f^{\prime \prime }g^{\prime }\theta^{\prime }+\xi^{2}g^{\prime \prime }g^{\prime }\theta^{\prime }\}-\frac{\left(n-1\right)}{2}(gg^{\prime }\theta^{\prime }+fg^{\prime }\theta^{\prime }+ff^{\prime }\theta^{\prime }+f^{\prime }g\theta^{\prime })+\frac{\left(n+1\right)}{2}\\ -(g^{2}\theta^{\prime \prime }+f^{2}\theta^{\prime \prime }+fg\theta^{\prime \prime })]=0, \end{array}$$ (14)

$$\begin{array}{l} \frac{1}{Sc}\varphi^{\prime \prime }+f\varphi^{\prime }+g\varphi^{\prime }+\gamma [\frac{(n-1{)}^{2}}{2(n+1)}\{\xi^{2}f^{\prime 2}\varphi^{\prime \prime }+\xi^{2}g^{\prime 2}\varphi^{\prime \prime }-\xi f^{\prime \prime }g^{\prime }\varphi^{\prime }-\xi g^{\prime \prime }g^{\prime }\varphi^{\prime }\\ +\xi^{2}f^{\prime \prime }g^{\prime }\varphi^{\prime }+\xi^{2}g^{\prime \prime }g^{\prime }\varphi^{\prime }\}-\frac{\left(n-1\right)}{2}(gg^{\prime }\varphi^{\prime }+fg^{\prime }\varphi^{\prime }+ff^{\prime }\varphi^{\prime }+f^{\prime }g\varphi^{\prime })+\frac{\left(n+1\right)}{2}\\ -\left(g^{2}\varphi^{\prime \prime }+f^{2}\varphi^{\prime \prime }+fg\varphi^{\prime \prime }\right)]=0, \end{array}$$ (15)

$$\begin{array}{l} f^{\prime }(\beta )=1,g^{\prime }(\beta )=1,f(\beta )=-\frac{2(n-1)\beta }{\left(n+1\right)},g(\beta )=0,\theta (\beta )=1,\varphi (\beta )=1\;\mathrm{at}\;\Lambda =\beta ,\\ f^{\prime }(\Lambda )\to 0,g^{\prime }(\Lambda )\to 0,\theta (\Lambda )\to 0,\varphi (\Lambda )\to 0\;\mathrm{as}\;\Lambda \to \infty . \end{array}$$ (16)

Here $\beta =A\sqrt{\frac{(n+1)c}{2\nu_{f}}}$ is the wall thickness parameter.

Writing

f(Λ)=f(ξ−β)=F(ξ), (17)

g(Λ)=g(ξ−β)=G(ξ), (18)

θ(Λ)=θ(ξ−β)=Θ(ξ), (19)

φ(Λ)=φ(ξ−β)=Φ(ξ). (20)

Eqs (12–15) become:

$$\frac{1}{\left(1-\varphi {)}^{2.5}(1-\varphi +\frac{\rho_{s}}{\rho_{f}}\varphi \right)}F^{\prime \prime \prime }+FF^{\prime \prime }+GF^{\prime \prime }-\left(\frac{2n}{n+1}\right)F^{\prime 2}-\left(\frac{2n}{n+1}\right)F^{\prime }G^{\prime }+\frac{4\lambda }{n+1}G^{\prime }=0,$$ (21)

$$\frac{1}{\left(1-\varphi {)}^{2.5}(1-\varphi +\frac{\rho_{s}}{\rho_{f}}\varphi \right)}G^{\prime \prime \prime }+FG^{\prime \prime }+GG^{\prime \prime }-\left(\frac{2n}{n+1}\right)G^{\prime 2}-\left(\frac{2n}{n+1}\right)F^{\prime }G^{\prime }-\frac{4\lambda }{n+1}F^{\prime }=0,$$ (22)

$$\begin{array}{l} \frac{1}{Pr}\frac{k_{nf}}{k_{f}}\frac{1}{\left(1-\varphi +\frac{(\rho c_{p{)}_{s}}}{(\rho c_{p{)}_{f}}}\varphi \right)}\Theta^{\prime \prime }+F\Theta^{\prime }+G\Theta^{\prime }+\delta [\frac{(n-1{)}^{2}}{2(n+1)}\{\xi^{2}{F^{\prime }}^{2}\Theta^{\prime \prime }+\xi^{2}{G^{\prime }}^{2}\Theta^{\prime \prime }-\xi F\prime \prime G\prime \Theta \prime \\ -\xi G^{\prime \prime }G^{\prime }\Theta^{\prime }+\xi^{2}F^{\prime \prime }G^{\prime }\Theta^{\prime }+\xi^{2}G^{\prime \prime }G^{\prime }\Theta^{\prime }\}-\frac{\left(n-1\right)}{2}(GG^{\prime }\Theta^{\prime }+FG^{\prime }\Theta^{\prime }+FF^{\prime }\Theta^{\prime }+F^{\prime }G\Theta^{\prime })+\frac{\left(n+1\right)}{2}\\ -\left(G^{2}\Theta^{\prime \prime }+F^{2}\Theta^{\prime \prime }+FG\Theta^{\prime \prime })\right]=0, \end{array}$$ (23)

$$\begin{array}{l} \frac{1}{Sc}\Phi^{\prime \prime }+F\Phi^{\prime }+G\Phi^{\prime }+\gamma [\frac{(n-1{)}^{2}}{2(n+1)}\{\xi^{2}F^{\prime 2}\Phi^{\prime \prime }+\xi^{2}G^{\prime 2}\Phi^{\prime \prime }-\xi F^{\prime \prime }G^{\prime }\Phi^{\prime }-\xi G^{\prime \prime }G^{\prime }\Phi^{\prime }\\ +\xi^{2}F^{\prime \prime }G^{\prime }\Phi^{\prime }+\xi^{2}G^{\prime \prime }G^{\prime }\Phi^{\prime }\}-\frac{\left(n-1\right)}{2}(GG^{\prime }\Phi^{\prime }+FG^{\prime }\Phi^{\prime }+FF^{\prime }\Phi^{\prime }+F^{\prime }G\Phi \Theta^{\prime })\\ +\frac{\left(n+1\right)}{2}(G^{2}\Phi^{\prime \prime }+F^{2}\Phi^{\prime \prime }+FG\Phi^{\prime \prime })]=0, \end{array}$$ (24)

with boundary conditions

$$\begin{array}{l} F^{\prime }(0)=1,G^{\prime }(0)=1,F(0)=-\frac{2(n-1)\beta }{\left(n+1\right)},G(0)=0,\Theta (0)=1,\Phi (0)=1,\\ F^{\prime }(\infty )\to 0,G^{\prime }(\infty )\to 0,\Theta (\infty )\to 0,\Phi (\infty )\to 0. \end{array}$$ (25)

Here $\mathrm{Pr}=\frac{\nu_{f}(\rho c_{p}{)}_{f}}{k_{f}}$ stands for Prandtl number, $\lambda =\Omega (x+y{)}^{n-1}/c$ denotes rotation parameter, $\delta =\lambda_{E}c(x+y{)}^{n-1}$ denotes the thermal relaxation time and $\gamma =\lambda_{C}c(x+y{)}^{n-1}$ denotes the mass relaxation time.

Skin friction coefficients along the *x*− and *y*− directions are defined as follows:

$$C_{fx}=\frac{\tau_{wx}}{\rho_{f}u_{w}^{2}},C_{fy}=\frac{\tau_{wy}}{\rho_{f}v_{w}^{2}},$$ (26)

where the surface shear stresses *τ*_*wx*_ and *τ*_*wy*_ along *x*− and *y*− directions are

$$\tau_{wx}={\mu_{nf}\frac{\partial u}{\partial z}|}_{z=0},\tau_{wy}={\mu_{nf}\frac{\partial v}{\partial z}|}_{z=0}.$$ (27)

Dimensionless skin friction coefficients are

Cfx(Rex)1/2=1(1−φ)2.5f″(0),Cfy(Rey)1/2=1β3/2(1−φ)2.5g″(0), (28)

where (Rex)1/2=xc/νf and (Rey)1/2=yc/νf denote the local Reynolds number.

## 3. Results and discussion

In this study, the nonlinear and coupled Eqs (21)-(24) with boundary conditions (25) are solved numerically using Runge-Kutta-4 with shooting method for different values of parameters. Tables 1 and 2 are prepared for the skin friction coefficient in *x-*, *y-* directions for various values of *n*, *λ*, *β* and *ϕ*.

**Table 1:** Thermophysical properties of the nanoparticles and base fluid (water).

Properties	Sliver (Ag)	*Copper(Cu)*	Water (Pr = 6.2)
*ρ* (kg/m^3^)	10,500	8933	997.1
*C*_*p*_ (J/kg K)	235	385	4179
*k* (W/m K)	429	401	0.613

**Table 2:** Variation of skin friction coefficient (Rex1/2Cfx) with different values of *ϕ*, *λ*, *n* and *β*.

		*n* = 0				*n* = 1			
	*ϕ*	*λ* = 0.2		*λ* = 0.5		*λ* = 0.2		*λ* = 0.5	
*Ag-water*		*β* = 0.5	*β* = 1	*β* = 0.5	*β* = 1	*β* = 0.5	*β* = 1	*β* = 0.5	*β* = 1
	0.05	-1.78589	-3.10892	- 1.47080	- 2.76750	- 1.62147	- 1.62146	- 1.38789	- 1.38789
	0.1	-2.31237	-4.08215	-1.91915	-3.66412	-1.99524	-1.99524	-1.70783	-1.70783
	0.2	-3.39246	-6.04604	-2.83129	-5.45873	-2.81992	-2.81991	-2.41371	-2.41371
*Cu-water*	0.05	-1.70536	-2.95248	-1.40042	-2.61996	-1.57773	-1.57773	-1.35046	-1.35046
	0.1	-2.15235	-3.76926	-1.77833	-3.36705	-1.91329	-1.91329	-1.63768	-1.63768
	0.2	-3.07363	-5.42017	-2.54938	-4.86193	-3.07364	-5.42018	-2.54939	-4.86193

Figs 2–20 are arranged to investigate the characteristics of nondimensional velocities *f*′(*ξ*), and *g*′(*ξ*), temperature *θ*(*ξ*), concentration *Φ*(*ξ*), and skin friction coefficient for various values of emerging parameters such as: solid volume fraction *ϕ*, velocity power index *n*, wall thickness parameter *β*, rotation parameter *λ* and thermal relaxation time parameter *δ*.

**Fig 2:** Effect of *n*, *ϕ* on *f*′(*ξ*).

**Fig 3:** Effect of *n*, *ϕ* on *g*′(*ξ*).

**Fig 4:** Effect of *λ*, *ϕ* on *f*′(*ξ*).

**Fig 5:** Effect of *λ*, *ϕ* on *g*′(*ξ*).

**Fig 6:** Effect of *β*, *ϕ* on *f*′(*ξ*).

**Fig 7:** Effect of *β*, *ϕ* on *g*′(*ξ*).

**Fig 8:** Effect of *n*, *ϕ* on *θ*(*ξ*).

**Fig 9:** Effect of *λ*, *ϕ* on *θ*(*ξ*).

**Fig 10:** Effect of *β*, *ϕ* on *θ*(*ξ*).

**Fig 11:** Effect of *δ*, *ϕ* on *θ*(*ξ*).

**Fig 12:** Effect of *n*, *ϕ* on *Φ*(*ξ*).

**Fig 13:** Effect of *λ*, *ϕ* on *Φ*(*ξ*).

**Fig 14:** Effect of *β*, *ϕ* on *Φ*(*ξ*).

**Fig 15:** Effect of *γ*, *ϕ* on *Φ*(*ξ*).

**Fig 16:** Effect of Sc, φ on *Φ*(*ξ*).

**Fig 17:** Effect of *λ*, *β*, *ϕ* on (Re_x_)^1/2^C_fx_.

**Fig 18:** Effect of *λ*, *β*, *ϕ* on (Re_y_)^1/2^C_fy_.

**Fig 19:** Streamlines for different values of nanoparticles volume fraction *ϕ* at *λ* = *n* = *β* = 3.

**Fig 20:** Isotherms for different values of nanoparticles volume fraction *ϕ* at *λ* = *n* = *β* = 3, *δ* = *γ* = 2.

Figs 2(A), 2(B) and 3(A), 3(B) show the impact of various values of *n* and *ϕ* on velocities along *x-* and *y-* axis respectively. We analyzed that the velocity profiles upsurge (in both directions) with enhancing the values of *n* for both *Ag*- and *Cu*-water while an opposite trend is noticed for solid volume fraction parameter in *x-* and *y-*directions. Because when nanoparticles volume fraction increases, friction enhances which decreases the fluid flow. Characteristics of *λ* and *ϕ* on velocity field are presented in Figs 4(A), 4(B) and 5(A), 5(B) along *x-* and *y-* axis respectively. Here, the fluid velocity in both directions peters out with the augmented values of *λ* and *ϕ*. Physically, the higher value of rotation parameter corresponds to lower stretching rates (along *x-*direction) compared to the rotation rate. Moreover, it is also observed that the momentum boundary layer thickness reduced for *Cu*-water is slightly quicker than *Ag*-water case. Figs 6(A), 6(B) and 7(A), 7(B) illustrate the effects of *β* and *ϕ* on velocity profile. The growth in the fluid velocity is observed for solid volume fraction parameter while the larger values of wall thickness parameter correspond to small deformation due to stretching of wall and hence the velocity peters out in *x-* and *y-*directions.

Fig 8(A) and 8(B) shows the impact of nanoparticles volume fraction *ϕ* and velocity power index *n* on temperature profile *θ*(*ξ*). An enhancement is observed for temperature profile *θ*(*ξ*) when nanoparticles volume fraction *ϕ* is increased. Physically, the thermal conductivity upsurges for higher value of the solid volume fraction parameter and consequently, fluid temperature increase. For nanoparticles volume fraction, the temperature of nanofluid containing copper nanoparticles was lower than that of containing silver nanoparticles. It is because the thermal conductivity of silver nanoparticles is high so the thickness of related boundary layer of Ag–water is greater than that of Cu–water nanofluid. It is further noticed that the thermal boundary layer is more thickens for an increasing value of velocity power index *n*. Fig 9(A) and 9(B) depicts the impact of *λ* and *ϕ* on the non-dimensional temperature field *θ*(*ξ*). It has been noticed that the temperature and thermal boundary layer escalate with increasing values of *λ* and *ϕ*. Because when rotation parameter is increased, the fluid resistivity increases which as a result enhances the fluid temperature. Fig 10(A) and 10(B) illustrate the influence of *β* and *ϕ* on temperature field *θ*(*ξ*). The growth in the fluid temperature is noticeably seen for solid volume fraction parameter while the larger values of wall thickness parameter upsurge the fluid temperature within boundary layer so that the related thermal layer become more thickens. Impact of thermal relaxation time parameter *δ* and *ϕ* on the temperature filed *θ*(*ξ*) is sketched in Fig 11(A) and 11(B). For *Ag*- and *Cu*-water, the temperature and related thermal layer thickness escalating with larger values of *δ*. As thermal relaxation parameter enlarges, the penetration depth of temperature decreases which enhances the temperature.

The effects of *n* and *ϕ* on concentration *Φ*(*ξ*) is discussed in Fig 12(A) and 12(B). Large values of *n* and *ϕ* give rise into the nanoparticles concentration *Φ*(*ξ*) and the related boundary layer thickness. Fig 13(A) and 13(B) is presented to characterize the behavior of *λ* and *ϕ* on the nanoparticles concentration *Φ*(*ξ*). From this Fig 1 can see that an increment in *λ* leads to higher nanoparticles concentration. As rotation parameter enhances resistivity which enhances the fluid concentration. Fig 14(A) and 14(B) shows the effects of *β* and *ϕ* on nanoparticles concentration *Φ*(*ξ*). The decline in the nanoparticles concentration is noticeably seen for the larger values of wall thickness parameter while an increase in solid volume fraction parameter cause the rise in nanoparticles concentration and the related thermal layer thickness. Impact of the mass relaxation time parameter *γ* and *ϕ* on nanoparticles concentration *Φ*(*ξ*) is sketched in Fig 15(A) and 15(B). As mass relaxation time is directly proportion to the parameter λ_c,_ the curves tend to move in the vicinity of stretching boundary and concentration and solutal boundary layer thickness escalating with larger values of *γ*. Fig 16(A) and 16(B) shows that larger Schmidt number *Sc* results in thinner concentration boundary layer as larger Schmidt number *Sc* fluid has higher concentration diffusivity and nanoparticles concentration peter out for larger values of Schmidt number.

The skin friction factors on (Re_x_)^1/2^C_fx_ and (Re_y_)^1/2^C_fy_ against the volume fraction *ϕ* and for different values of *β* and *λ* is illustrating in Figs 17(A), 17(B) and 18(A) and 18(B). The values of skin friction coefficients (Re_x_)^1/2^C_fx_ and (Re_y_)^1/2^C_fy_ are negative since the fluid applies stress on the stretching wall (that causes the flow). Clearly, the magnitudes of (Re_x_)^1/2^C_fx_ and (Re_y_)^1/2^C_fy_ are an increasing function of *ϕ*. This fact can also be verified from the tabular values of skin friction factors (Re_x_)^1/2^C_fx_ and (Re_y_)^1/2^C_fy_ as presented in Tables 2 and 3 while Thermophysical properties of nanoparticles and water are given in Table 1.

**Table 3:** Variation of skin friction coefficient (Rey1/2Cfy) with different values of *ϕ*, *λ*, *n* and *β*.

		*n* = 0				*n* = 1			
	*ϕ*	*λ* = 0.2		*λ* = 0.5		*λ* = 0.2		*λ* = 0.5	
*Ag-water*		*β* = 0.5	*β* = 1	*β* = 0.5	*β* = 1	*β* = 0.5	*β* = 1	*β* = 0.5	*β* = 1
	0.05	-7.62249	-3.79191	- 9.78189	- 4.37888	- 5.87440	- 2.07691	- 6.94077	- 2.4539
	0.1	-9.63955	-4.88781	-12.2536	-5.57904	-7.22856	-2.55568	-8.54075	-3.01961
	0.2	-13.9066	-7.14930	-17.5537	-8.09412	-10.2162	-3.61199	-12.0708	-4.26767
*Cu-water*	0.05	-7.34383	-3.62733	-9.45701	-4.20753	5.71596	-2.02089	-6.75357	-2.38775
	0.1	-9.09617	-4.56124	-11.6274	-5.24149	-6.93163	-2.45070	-8.18992	-2.89557
	0.2	-12.8371	-6.49921	-16.3309	-7.42514	-12.8371	-6.49921	-16.3309	-7.42514

The streamlines of the current analysis are drawn in Fig 19 for two different values of solid volume fractions (*ϕ* = 0,0.1). It is exposed that with the presence of solid volume fraction the rotating effects is more strengthen. The isotherms behavior outlines along the surface for two values of solid volume fractions have been explored in Fig 20. From the first plot of the isotherms, it is evidently seen that the isotherms are closed to small *ξ* and very closed too in the second plot in the case of *ϕ* = 0.1. This leads us to the result that for *ϕ* = 0.1, the accumulation of isotherms around the dimensionless variable *ξ* is increased.

Fig 21(A) and 21(B) presents −*θ*′(0) as a function of nanoparticles volume fraction φ for both *Ag*- and *Cu*-water against different values of wall thickness parameter β and rotation parameter λ. There is an increase in −*θ*′(0) for larger wall thickness and rotation parameters. Also, magnitude of −*θ*′(0) is inversely proportional to φ. Variations of −Φ′(0) via nanoparticles volume fraction φ for different values of Schmidt number Sc and mass relaxation time parameter γ are depicted in Fig 22(A) and 22(B). There is an increase in the magnitude of −Φ′(0) when Sc is increased. While magnitude of −Φ′(0) has inverse relationship with γ and φ.

**Fig 21:** Effect of *ϕ*, *β*, *λ* on −*θ*′(0).

**Fig 22:** Effect of *ϕ*, *γ*, *Sc* on −Φ′(0).

In Table 4 we compared the results of *f*″(0) and *g*″(0) with existing literature in limiting sense. It is observed that obtained results are in good agreement with present findings.

**Table 4:** Comparison of *f*″(0) and *g*″(0) for value of n when other parameters are zero.

*n* = 1	Khan et al. [50]		Present result	
	*f*″(0)	*g*″(0)	*f*″(0)	*g*″(0)
	-1.414214	-1.414214	-1.414214	-1.414214

## 4. Conclusions

The applications of stretching sheet are not only limited to industry but also finds its place in the geological studies where the fluid flows over submerged tectonic plate in rotating condition. Motivated by such applications the present article addresses three-dimensional rotational flow of nanofluid over nonlinearly stretching sheet of variable thickness. Tiwari and Das model is taken for nanofluid. The energy and concentration equations are modeled by incorporating CC-heat and mass flux effects. The mathematically modeled non-linear system of equations is solved with RK-4 cum shooting technique. The numerical and graphical outcomes for flow, energy and mass transport are obtained for various values of pertinent parameters. The computational investigation leads to some important results outlined as below:

■ Fluid flow, heat and mass are increasing functions of power law index.
■ Hydrodynamic boundary layer thickness is reduced due to larger nanoparticles volume fraction and rotation parameter
■ Thermal field *θ*(*ξ*) and the related boundary layer get increased due to the inclusion of rotation, nanoparticles volume fraction and thermal relaxation time.
■ Augmented *β* and *Sc* yield deescalated concentration *Φ*(*ξ*) and the related boundary layer.
■ Rise in *β* improves viscous drag force, from stretching surface, however, declines the same for solid volume fraction parameter *ϕ*.
■ For *ϕ* = 0.1, the accumulation of isotherms around the dimensionless variable *ξ* is increased.

## Abbreviations

u, v, w: Velocity components along x-, y- and z- axis (m/s)
T: Temperature (K
T_w_: Wall temperature (K)
T_∞_: Ambient fluid temperature (K)
C: Fluid concentration
C_w_: Wall concentration
C_∞_: Ambient fluid concentration
u_w_: Fluid wall velocity along x-axis (m/s
v_w_: Fluid wall velocity along y-axis (m/s)
k: Thermal conductivity (WK^-1^m^-1^)
C_p_: Specific heat (m^2^s^-2^
c: Stretching rate constant
n: Wall thickness parameter (m)
D: Diffusion coefficient
Pr: Prandtl number
C_f_: Local skin friction coefficient Subscripts
Re: Local Reynolds number
Greek symbols: λ_E_: Heat relaxation time (s)
λ_C_: Mass relaxation time (s)
Ω: Angular velocity (rad.s^-1^)
ν: Kinematic viscosity (m^2^s^-1^)
ρ: Density (kgm-3)
μ: Dynamic viscosity (kgm^-2^s^-1^)
α: Thermal diffusivity (m^2^s^-1^
φ: Nanoparticles volume fraction
Ʌ: ξ Transformed coordinate
β: Wall thickness parameter
λ: Rotation parameter
δ: Thermal relaxation time
γ: Mass relaxation time
τ_w_: Wall shear stress
Subscripts: s, f, nf: denotes nano-solid particles, base fluid and nanofluid
